# Logistic Regression Analysis of Clinical Characteristics for Differentiation of Chronic Obstructive Pulmonary Disease Severity

**DOI:** 10.1155/2023/5945191

**Published:** 2023-02-08

**Authors:** Shuaixing Guo

**Affiliations:** Changzhen Community Service Center, Shenzhen Hospital, University of Chinese Academy of Sciences, Shenzhen, China

## Abstract

**Background:**

This study aimed to investigate the predictive value of general clinical data, blood test indexes, and ventilation function test indexes on the severity of chronic obstructive pulmonary disease (COPD).

**Methods:**

A total of 141 clinical characteristics of COPD patients admitted to our hospital were collected. A mild-to-moderate group and a severe group were classified depending on the severity of COPD, and their baseline data were compared. The predictive factors of severe COPD were analyzed by univariate and multivariate logistic regression, and the nomogram model of severe COPD was constructed. The clinical variables, including gender, height, weight, body mass index (BMI), age, course, diabetes, hypertension, smoking history, WBC, NEUT, lymphocyte count (LY), MONO, eosinophil count (EOS), PLT, mean platelet volume (MPV), platelet distribution width (PDW), partial pressure of oxygen (PaO_2_), and PaCO_2_, were collected.

**Results:**

There were 67 mild-to-moderate COPD patients and 74 severe COPD patients in this study cohort. Severe COPD had a higher white blood cell count (WBC), neutrophil count (NEUT), monocyte count (MONO), platelet count (PLT), neutrophil to lymphocyte ratio (NLR), and a lower partial pressure of carbon dioxide (PaCO_2_). Univariate logistic regression analysis showed that WBC, NEUT, MONO, PLT, and NLR were contributing factors of severe COPD, while PaCO_2_ was an unfavorable factor of severe COPD. Enter, forward, backward, and stepwise multivariate logistic regression analyses all showed that NEUT and PLT were independent contributing factors to severe COPD. Moreover, the nomogram model had good predictive ability, with an area under the curve (AUC) of the receiver operating characteristic (ROC) curve being 0.881. Good calibration and clinical utility were validated through the calibration plot and the decision curve analysis (DCA) plot, respectively.

**Conclusion:**

The severity of COPD was correlated with NEUT and PLT, and the nomogram model based on these factors had good predictive performance.

## 1. Introduction

Chronic obstructive pulmonary disease (COPD), one of the most common respiratory diseases, is characterized by persistent airflow limitation and multiple complications [1]. Its high morbidity, hospitalization, disability, and mortality rates impose a serious economic burden on families and society [2]. According to the 2010 Global Burden of Disease Study, COPD was estimated to be the third leading cause of life expectancy loss in China [3]. The latest statistics from the World Health Organization show that moderate or severe COPD affects approximately 65 million people worldwide and that COPD will be the third leading cause of death worldwide by 2030. Correct assessment of disease severity and optimal treatment are essential for better clinical and socioeconomic outcomes for COPD patients [4].

The Global Initiative for Chronic Obstructive Lung Disease (GOLD) guidelines state that forced expiratory volume in one second (FEV1) and forced vital capacity (FVC) can be used as valid indicators of lung function [5]. Based on these two indicators, the condition can be classified into four classes. However, pulmonary function testing is a test that relies on patient-physician cooperation, and test results depend on measurement technique and personal factors. A related study has shown that nearly half of the pulmonary function tests have unreliable data due to failure to complete the test effectively, causing some disturbance in treatment [6]. Therefore, there is an urgent clinical need to find indicators for the assessment of COPD severity.

Recent studies have found that C-reactive protein (CRP), procalcitonin (PCT), interleukin-6 (IL-6), IL-8, tumor necrosis factor-*α* (TNF-*α*), and other inflammatory indicators are all associated with the development of COPD [7, 8]. However, each of these indicators has its own advantages and disadvantages. For example, CRP and PCT assays are economical and convenient but susceptible to a variety of factors. IL-6, IL-8, and TNF-*α* are highly sensitive but more expensive to detect. As emerging inflammatory indicators, the neutrophil-to-lymphocyte ratio (NLR), platelet-to-lymphocyte ratio (PLR), and lymphocyte-to-monocyte ratio (LMR) are derived from the complete blood count and all are related to the degree of inflammation and clinical symptoms of COPD [9, 10]. Elevated NLR levels have been reported in thyroid conditions [11], irritable bowel disease [12], COVID-19 infection [13], diabetes mellitus [14], and thyroiditis [15]. However, the use of blood count indicators and their derivatives in the classification of COPD severity has rarely been reported.

To accurately classify and effectively treat COPD patients, many scholars have investigated machine learning algorithms to assist clinical decision-making [16, 17]. This study proposes a method for severity classification assessment and risk prediction of COPD patients' conditions using common clinical information when lung function tests are not available and to assist physicians in patient classification based on the severity of different COPD patients.

## 2. Methods

### 2.1. Clinical Data Collection

141 COPD patients treated in our hospital were included, with 67 patients having mild-to-moderate and 74 patients having severe. The severity of COPD was clinically assessed in these patients. The clinical variables were collected, including gender, height, weight, body mass index (BMI), age, course, diabetes, hypertension, smoking history, WBC, NEUT, lymphocyte count (LY), MONO, eosinophil count (EOS), PLT, mean platelet volume (MPV), platelet distribution width (PDW), partial pressure of oxygen (PaO_2_), and PaCO_2_. Besides, three inflammation indicators, including NLR, platelets and lymphocytes ratio (PLR), and lymphocytes to monocytes ratio (LMR), were calculated. All patients signed the consent form, and this study has been approved by the Ethical Committee of the University of Chinese Academy of Sciences Shenzhen Hospital.

### 2.2. Statistical Analysis

R4.2.0 was used for data processing. Categorical data were expressed as frequencies and percentages and compared by the chi-squared test between groups. Measurement data were tested for normality, and then normally distributed measurement data were expressed as mean ± standard deviation and compared by a *t*-test between groups. Nonnormally distributed measurement data were expressed as median (interquartile range) and compared by the Wilcoxon rank sum test between groups. The difference was considered statistically significant at *P*  <  0.05. A logistic regression analysis was used to examine the influencing factors predicting COPD severity. Significant predictive factors in the univariate logistic regression analysis were selected for the multivariate logistic regression analysis with enter, forward, backward, or stepwise methods, respectively. Then, a nomogram model was developed based on independent predictive factors with the rms package of R. The discrimination of the nomogram model was estimated by the receiver operating characteristic (ROC) curve. The calibration was validated by a calibration plot using the bootstrap method with 50 repetitions using the caret package. The clinical utility was analyzed by a decision curve analysis (DCA) plot using the rmda package. For internal validation, 5-fold cross-validation was applied.

## 3. Results

### 3.1. Baseline Data Comparison

This study included 141 COPD patients, with 67 having mild-to-moderate COPD and 74 having severe COPD (Table 1). In severe COPD, WBC (Figure 1(a)), NEUT (Figure 1(b)), MONO (Figure 1(c)), PLT (Figure 1(d)), and NLR (Figure 1(e)) were higher than those in mild-to-moderate COPD, while PaCO_2_ (Figure 1(f)) was lower than that in mild-to-moderate COPD.

### 3.2. Logistic Regression Analysis of Influencing Factors with Severity in COPD Patients

Through univariate logistic regression analysis on all clinical variables, we identified WBC, NEUT, MONO, PLT, NLR, and PaCO_2_ as influencing factors of severe COPD (Table 2). Furthermore, through multivariate logistic regression analysis with enter (Figure 2), forward (Figure 3), backward (Figure 4), and stepwise (Figure 5) methods, we identified NEUT and PLT as independent predictive factors.

### 3.3. Nomogram Model for Predicting COPD Severity

Based on NEUT and PLT, we constructed a nomogram model for predicting COPD severity (Figure 6). The AUC of the ROC curve was 0.881, indicating good discrimination of the nomogram model (Figure 7(a)). Besides, the predicted probability was close to the observed probability in the calibration plot, suggesting good calibration of the nomogram model (Figure 7(b)). Furthermore, the DCA curve implied good clinical utility of the nomogram model (Figure 7(c)). For internal validation, 5-fold cross-validation was applied, and the mean AUC of the training sets was 0.87492 (Table 3).

## 4. Discussion

There is some difficulty in completing normal lung function tests for severe COPD patients, and there is significant heterogeneity in clinical manifestations and disease progression between patients with different severity levels, so it is important to classify COPD patients and target therapy. Machine learning provides a powerful tool for the classification and prediction of severity in COPD patients. In this study, we identified 2 independent risk factors for severe COPD, including NEUT and PLT, by univariate and multifactorial logistic regression. Based on these, the nomogram model had good performance.

Although several biochemical markers have been investigated as predictors of COPD outcome, their measurement is usually time- and resource-intensive [18]. Relatively simple biomarkers of inflammation calculated from routine complete blood count tests may also predict COPD progression and outcome [19]. Chronic inflammation is an important pathogenesis of COPD, involving a complex interaction of various immune-related cells (including neutrophils and lymphocytes), which may lead to persistent airway damage and lung parenchymal destruction, which in turn decreases lung function and immune function. In the long run, COPD patients are prone to acute exacerbations of their disease due to various external triggers. NEUT is a risk indicator for mortality in COPD patients [20]. A variety of activated immune cells, mainly NEUs, result in the release of reactive oxygen species, causing a cascade of inflammatory responses [21]. In addition, activated neutrophils can produce not only other important inflammatory mediators such as proteases, matrix metalloproteinases, and myeloperoxidase [22], leading to lung parenchymal destruction and emphysematous changes, but also cytokines, enzymes, adhesion molecules, and growth factors, contributing to the recruitment of inflammatory cells to the airways [23]. The abovementioned pathological process leads to an increased local and systemic inflammatory response, which aggravates lung tissue and vascular damage and even induces respiratory failure in severe cases. Besides, PLT is reported as a diagnostic marker for the development of COPD [24]. In this study, we found that the NEUT and PLT levels gradually increase as COPD disease worsens and are risk factors for COPD severity.

The present study has some limitations. First, this study only analyzed the relationship between general clinical data, routine blood indicators, PaO_2_, PaCO_2_, and COPD severity; further analysis of the relationship between other test indicators and COPD severity is still needed. Second, this study is a single-center retrospective study, and the results can only indicate that high NEUTs and PLTs are risk factors for severe COPD. A more extensive prospective, multicenter clinical trial with a more detailed stratification of the study population is necessary to further confirm the value of NEUTs and PLTs in COPD.

In summary, both NEUT and PLT are independent risk factors for severe COPD, and their combined application has a high predictive value for COPD severity.

## Figures and Tables

**Figure 1:** The difference in clinical characteristics, including WBC (a), NEUT (b), MONO (c), PLT (d), NLR (e), and PaCO_2_ (f), between mild-to-moderate and severe COPD groups.

**Figure 2:** Multivariate logistic regression analysis with enter method.

**Figure 3:** Multivariate logistic regression analysis with forward method.

**Figure 4:** Multivariate logistic regression analysis with backward method.

**Figure 5:** Multivariate logistic regression analysis with stepwise method.

**Figure 6:** Nomogram model based on independent predictive factors for COPD severity.

**Figure 7:** The performance of the nomogram model. (a) ROC curve. (b) Calibration curve. (c) DCA curve.

**Table 1:** Comparison of clinical characteristics between the mild-to-moderate group and the severe group in COPD patients.

Characteristics	Mild-to-moderate	Severe	*p*
*n*	67	74	
Gender, *n* (%)			
Female	16 (11.3%)	11 (7.8%)	0.252
Male	51 (36.2%)	63 (44.7%)	
Diabetes, *n* (%)			
No	59 (41.8%)	70 (49.6%)	0.277
Yes	8 (5.7%)	4 (2.8%)	
Hypertension, *n* (%)			
No	39 (27.7%)	38 (27%)	0.517
Yes	28 (19.9%)	36 (25.5%)	
Smoking history, *n* (%)			
No	24 (17%)	25 (17.7%)	0.939
Yes	43 (30.5%)	49 (34.8%)	
Height (cm), median (IQR)	167 (161.5, 170)	168 (164.25, 171)	0.161
Weight (kg), mean ± SD	58.94 ± 7.4	58.29 ± 9.5	0.656
BMI(kg/m^2^), median (IQR)	21.67 (19.95, 22.76)	20.99 (19.39, 22.68)	0.131
Age (year), median (IQR)	78 (70, 82)	74 (65.25, 81)	0.145
Course (year), median (IQR)	3 (0, 10)	3 (0.25, 8.75)	0.745
WBC (10^9^/L), median (IQR)	6.64 (5.56, 7.38)	10.19 (8.32, 11.67)	**<0.001** ^*∗∗∗*^
NEUT (10^9^/L), median (IQR)	4.65 (3.62, 5.48)	7.96 (6.02, 9.82)	**<0.001** ^*∗∗∗*^
LY (10^9^/L), median (IQR)	1.02 (0.66, 1.56)	1.19 (0.77, 1.63)	0.347
MONO (10^9^/L), median (IQR)	0.51 (0.41, 0.61)	0.62 (0.46, 0.82)	**0.006** ^*∗∗*^
EOS (10^9^/L), median (IQR)	0.09 (0.03, 0.22)	0.12 (0.02, 0.25)	0.988
PLT (10^9^/L), median (IQR)	181 (148, 218)	234 (180.75, 302)	**<0.001** ^*∗∗∗*^
MPV (fL), mean ± SD	9.15 ± 0.98	9.06 ± 1.17	0.630
PDW (%), median (IQR)	16 (15.7, 16.3)	16 (15.7, 16.3)	0.828
NLR, median (IQR)	4.21 (2.53, 6.15)	6.34 (3.56, 13.62)	**<0.001** ^*∗∗∗*^
PLR, median (IQR)	167.71 (116.07, 255.48)	205.2 (136.29, 305.16)	0.086
LMR, median (IQR)	1.88 (1.51, 3.39)	1.96 (1.25, 3.01)	0.331
PaO_2_ (mmHg), median (IQR)	78 (67.05, 95.4)	74.7 (63.68, 95.55)	0.668
PaCO_2_ (mmHg), median (IQR)	60.1 (47.55, 76.65)	48.25 (42.85, 59.45)	**0.002** ^*∗∗*^

^*∗∗*^=0.01,  ^*∗∗∗*^=<0.001.

**Table 2:** Results of univariate logistic regression analysis on influencing factors of severity in COPD patients.

Variables	*β*	SE	*z*	*p*	OR (95% CI)
Gender	−0.586	0.435	−1.348	0.178	0.55655 (0.23744, 1.30451)
Height	0.04	0.028	1.427	0.154	1.04085 (0.98515, 1.0997)
Weight	−0.009	0.020	−0.449	0.653	0.99112 (0.95327, 1.03047)
BMI	−0.08	0.062	−1.285	0.199	0.92327 (0.81739, 1.04287)
Age	−0.026	0.018	−1.436	0.151	0.9746 (0.94095, 1.00944)
Course	0.008	0.031	0.241	0.809	1.00755 (0.94788, 1.07097)
Diabetes	−0.864	0.637	−1.356	0.175	0.42143 (0.12084, 1.46978)
Hypertension	0.277	0.340	0.816	0.414	1.31955 (0.67796, 2.56829)
Smoking history	0.09	0.354	0.254	0.800	1.09395 (0.54658, 2.18949)
WBC	0.541	0.104	5.218	**0.000** ^*∗∗∗*^	1.71844 (1.40223, 2.10597)
NEUT	0.699	0.128	5.479	**0.000** ^*∗∗∗*^	2.01129 (1.56646, 2.58243)
LY	0.266	0.223	1.194	0.232	1.30453 (0.84329, 2.01806)
MONO	1.705	0.655	2.603	**0.009** ^*∗∗*^	5.50173 (1.52347, 19.86855)
EOS	0.341	0.720	0.474	0.636	1.40635 (0.34318, 5.76325)
PLT	0.012	0.003	4.073	**0.000** ^*∗∗∗*^	1.01214 (1.00628, 1.01803)
MPV	−0.076	0.157	−0.485	0.628	0.92687 (0.68203, 1.25961)
PDW	0.032	0.118	0.272	0.786	1.03255 (0.81963, 1.30079)
NLR	0.118	0.037	3.168	**0.002** ^*∗∗*^	1.12514 (1.04598, 1.2103)
PLR	0.002	0.001	1.322	0.186	1.0016 (0.99923, 1.00397)
LMR	−0.128	0.099	−1.296	0.195	0.87989 (0.72511, 1.06771)
PaO_2_	−0.007	0.010	−0.682	0.495	0.99315 (0.97372, 1.01297)
PaCO_2_	−0.03	0.010	−2.911	**0.004** ^*∗∗*^	0.97077 (0.95157, 0.99035)

^*∗∗*^=0.01,  ^*∗∗∗*^=<0.001.

**Table 3:** 5-fold cross-validation assessing the prediction capability of our model.

Fold	Cox-Snell *R*^2^	Nagelkerke *R*^2^	Accuracy	Precision	Recall	*F*_measure	AUC
1	0.83754	0.84152	0.89655	0.89474	0.94444	0.91892	0.94949
2	0.89234	0.89580	0.78571	0.80000	0.66667	0.72727	0.81771
3	0.90270	0.90608	0.75000	0.84615	0.68750	0.75862	0.81250
4	0.86202	0.86532	0.85714	0.90909	0.76923	0.83333	0.89744
5	0.89351	0.89687	0.82143	0.81250	0.86667	0.83871	0.89744
Mean	0.87762	0.88112	0.82217	0.85250	0.78690	0.81537	0.87492

## Data Availability

The data used to support this study are available from the corresponding author upon request.
